The article "Aberrant mannosylation profile and FTX/miR-342/ALG3-axis contribute to development of drug resistance in acute myeloid leukemia" was retracted in 2020. Reasons: duplicated data; concerns about the data.

# Aberrant mannosylation profile and FTX/miR-342/ALG3-axis contribute to development of drug resistance in acute myeloid leukemia

**DOI:** 10.1038/s41419-018-0706-7

**Published:** 2018-06-07

**Authors:** Bing Liu, Xiaolu Ma, Qianqian Liu, Yang Xiao, Shimeng Pan, Li Jia

**Affiliations:** 1 College of Laboratory Medicine, Dalian Medical University, Dalian, 116044 Liaoning Province China; 2 Department of Clinical Laboratory, the First Affiliated Hospital of Dalian Medical University, Dalian, 116011 Liaoning Province China

## Abstract

Drug-resistance is a major problem in acute myeloid leukemia (AML) chemotherapy. Aberrant changes in specific *N*-glycans have been observed in leukemia multidrug resistance (MDR). MicroRNAs (miRNAs) and long non coding RNAs (lncRNAs) act as key players in the development of AML resistance to chemotherapy. In the present study, the *N*-glycan profiles of membrane proteins were analyzed from adriamycin (ADR)-resistant U937/ADR cells and sensitive line U937 cells using mass spectrometry (MS). The composition profiling of high-mannose *N*-glycans differed in U937/ADR and U937 cell lines. Lectin microarray showed that the strong binding of membrane proteins was observed for MAN-M and ConA lectins, which were specific for mannose. These binding were also validated by flow cytometry. Importantly, the alteration of high-mannose *N*-glycan was further confirmed by detecting the enzyme level of ALG family. The altered level of ALG3 was found corresponding to the drug-resistant phenotype of AML cell lines both in vitro and in vivo. Mechanistically, miR-342 was found to be dysregulated and inversely correlated to ALG3 expression, targeting its 3′-UTR. LncRNA FTX was a direct target of miR-342 and positively modulated ALG3 expression by competitively binding miR-342 in AML cell lines. Functionally, we found that FTX directly interacted with miR-342 to regulate ALG3 expression and function, including ADR-resistant cell growth and apoptosis. The observation suggested that high-mannose *N*-glycans and mannosyltransferase ALG3 affected drug-resistance in AML cells. FTX/miR-342/ALG3 axis could potentially be used for the targets to overcome therapeutic resistance in AML.

## Introduction

Acute myeloid leukemia (AML) is a highly invasive hematopoietic system malignant disease, and characterized by the clonal proliferation of myeloid precursors^1^. Allogenic stem cell transplantation accompanied with conventional chemotherapy appears as effective way to improve the recovery rates and increase the complete response in AML patients. However, multi-drug resistance (MDR) and disease relapse remain the major obstacles in AML treatment. Most AML patients who respond to primary chemotherapy later still experience MDR and relapse^2^. Therefore, clarifying the potential molecular mechanism involved in MDR is critical for the effective treatment against AML.

The article "Aberrant mannosylation profile and FTX/miR-342/ALG3-axis contribute to development of drug resistance in acute myeloid leukemia" was retracted in 2020. Reasons: duplicated data; concerns about the data.

*N*-linked protein glycosylation is one of the most common posttranslational modifications, wherein *N*-glycans are involved in a variety of biochemical and cellular processes^3^. Altered glycosylation is the common feature of tumor cells, also exhibiting a key role in several physiological and pathological procession^4^. Tumor-associated glycans, differential expression of glycosyltransferases and their target proteins within the tumor cell have been studied as specific tumor markers and potential therapeutic targets^5–7^, demonstrating the key function in cancer cell growth metastasis^8^. Aberrant expression of several high-mannose type *N*-glycans has been described during cancer progression. The abundant high mannose glycans are altered in patients sera of breast cancer^9^. High-mannose glycans are highly abundant features in both colorectal cancer cells and tumor samples^10^. Based on glycobiology, the differential glycosylation patterns between cancer and healthy control emerge as promising targets for identifying the potential cancer biomarkers.

Non-coding RNAs (ncRNAs), which lack protein-coding potential, have been focused on investigating the prognostic markers of AML. The most widely recognized class of ncRNAs is microRNAs (miRNAs) and long noncoding RNAs (lncRNAs). MiRNAs are usually only 18–24 nucleotides long, which repress protein expression through inhibiting mRNA transcription. MiRNAs are also important regulators of hematopoiesis and altered expression of them can be associated with the pathogenesis of hematologic malignancies^11–13^. Studies have shown that miRNAs are involved in the development of resistance against chemotherapy in AML. MiR-181b has been proved to decrease significantly in human MDR leukemia cells and relapsed/refractory AML patient samples^14^. LncRNAs which are a heterogeneous class of transcripts longer than 200 nucleotides, show numerous functions in AML pathogenesis^15^. Dysregulated lncRNAs contribute to various cellular processes in AML, including proliferation, apoptosis or migration^16^ and have been associated with poor clinical outcome^17^. One of the well-studied lncRNA, Hox antisense intergenic RNA myeloid 1 (HOTAIRM1), reveals clinical prediction for conventional therapy resistance. High expression of HOTAIRM1 is associated with shorter OS and unsatisfactory leukemia-free survival^18^. Although lncRNAs and miRNAs have been identified to affect AML therapy resistance, the specific function of lncRNA-FTX that modulates MDR of AML by directly targeting miR-342 to regulate ALG3 is not well understood.

The article "Aberrant mannosylation profile and FTX/miR-342/ALG3-axis contribute to development of drug resistance in acute myeloid leukemia" was retracted in 2020. Reasons: duplicated data; concerns about the data.

In the present study, the expression pattern of *N*-glycan in AML cell lines were examined, and the increased expression of ALG3 in AML cell lines was positively correlated AML MDR. FTX as a competing endogenous RNA regulated ALG3 expression by sponging miR-342 in AML. Furthermore, the underlying mechanism involved in FTX/miR-342/ALG3-regulated drug resistance in AML cell lines was explored.

## Materials and methods

### Clinical samples and cell culture

We recruited 38 untreated AML patients from the First Affiliated Hospital of Dalian Medical University (Dalian, China) during Jan 2016 to Feb 2018. The patients were composed of 21 males and 17 females with age ranging from 15 to 68 years (median age of 39.4 years). Peripheral blood mononuclear cells (PBMC) of AML were purified by Ficoll density gradient separation (Sigma-Aldrich) and cultured in dishes to remove adherent cells. We divided the PBMC into two groups, AML/MDR and AML without MDR groups, according to the fluorescence intensity higher than 20% of P-gp. The P-gp positivity frequency was 60.5% (23 of 38) of AML patients. All experiments were approved by the Institutional Ethics Committee of the First Affiliated Hospital of Dalian Medical University (Ethics Reference NO: YJ-KY-FB-2016-45).

Two AML cell lines, U937 and THP-1 were obtained from the KeyGEN Company (Nanjing, China) and grown in RPMI 1640 medium (Gibco) supplemented with 10% fetal bovine serum (Gibco), 1% penicillin-streptomycin at 37 °C in the incubator contained 5% CO_2_. The adriamycin-resistant (ADR) sublines were established by adding adriamycin (ADR, Sigma) to the parental cell. ADR concentrations were from 1 to 5 mg/l for 6 months and the cells were namely U937/ADR (U/A) and THP-1/ADR (T/A), respectively. The MDR phenotype of resistant AML cell lines was maintained through continuously supplementing with 1.0 mg/L ADR.

### Mass spectrometric analysis

Membrane protein extract was measured by a CelLytic MEM Protein Extraction kit (Sigma). The Micro BCA Protein Assay kit (PIERCE, Rockford, IL) was utilized to detect the membrane protein concentration. Three 100 μg aliquots of lyophilized cell membrane protein were digested and dissolved in 25 mM ammonium bicarbonate at 37 °C for 18 h. The digest product was bearing a water bath at 85 °C for 5 min, and the N-linked oligosaccharides were released from peptides with PNGase F treatment after cooling. The *N*-glycans released from glycoproteins were purified by Oasis HLB cartridge (60 mg/3 ml; Waters) and then lyophilized.

*N*-glycan profiles were obtained on MALDI-TOF mass spectrometer (Bruker Corp., Billerica, MA, USA). The released *N*-glycans were first permethylated. The permethylated glycans (0.5 μL) were spotted on a MALDI plate and sodiated DHB was added. The experiments were finished with a 4800 Proteomics Analyzer (Applied Biosystems). All MS spectra were obtained from Na+adductions.

The article "Aberrant mannosylation profile and FTX/miR-342/ALG3-axis contribute to development of drug resistance in acute myeloid leukemia" was retracted in 2020. Reasons: duplicated data; concerns about the data.

### Lectin microarray analysis

The lectin microarray analysis was performed by BC Biotechnology Co., LTD (Guangzhou, China). Lectin microarrays were blocked for 3 h in 50 μM ethethanolamine in a borate buffer. The blocked slides were washed by PBS. Membrane protein extract (final concentration was 50 μg/ml) were probed on the lectin microarray and incubated for overnight at 4 °C. The slides were then washed thrice with PBS and incubated with Cy3-streptavidin at 1 μg/ml. The slides were washed on a shaker for 5 min, air-dried, and scanned by a GenePix 4200A scanner. GenePix Pro 6.0 Software (Molecular Devices, Sunnyval, CA, USA) was used to analyze the fluorescence intensity of each spot. Lectins that showed signal intensity of higher than to three standard deviations above background were determined as positive signals.

### Quantitative real-time PCR

Total RNA was isolated from PBMC samples and AML cell lines by Trizol reagent (Invitrogen, USA). Using a PrimeScript™ RT reagent Kit (TaKaRa), the first strand cDNA was synthesized. The cDNA was amplifed by SYBR Premix Ex Taq™ II (TaKaRa). MiR-342 was normalized to U6, lncRNA FTX and ALG mRNA data were normalized to GAPDH. The relative expression of genes to internal control was calculated using the 2-ΔΔCT method. The sequences of the primers were shown in Table S1. All reactions were performed in triplicate.

### Western blot

In total 20 µg protein extract were separated on 10% SDS–PAGE and transferred to polyvinylidene difluoride transfer membranes. In total 5% skimmed milk was used to blocked the membrane. Then the membrane was incubated with the primary antibody ALG3 (1/250 diluted; Abcam, ab151211, Cambridge, UK) on a shaker at 4 °C for 12 h. The membrane was incubated with horseradish peroxidase-conjugated secondary antibody (rabbit IgG, 1/1000 diluted; UK). GAPDH antibody (1/200 diluted; Santa Cruz Biotech) was used as control. The bands were detected by ECL Western blot kit (Amersham Biosciences, UK) and analyzed by LabWorks (TM ver4.6, UVP, BioImaging systems).

### Flow cytometry (FCM) analysis

The apoptosis assay was performed using Annexin-V-FITC apoptosis kit (BD, Franklin Lakes, NJ, USA). Apoptosis rate of cells was analyzed by FACS Calibur flow cytometer (Becton-Dickinson, CA, USA), detecting the fluorescence of at least 10,000 cells each sample.

Cells were stained with the FITC-MNA-M, FITC-ConA and FITC-AAL lectins at a final concentration of 10 μg/ml in the dark. The labeled cells were resuspended in PBS and analyzed by FACS Calibur flow cytometer. Fluorescence intensity was measured by Cell Quest software. Each experiment was repeated in triplicate.

The article "Aberrant mannosylation profile and FTX/miR-342/ALG3-axis contribute to development of drug resistance in acute myeloid leukemia" was retracted in 2020. Reasons: duplicated data; concerns about the data.

### In vitro drug susceptibility assay

Drug susceptibility was measured using cell counting kit-8 (CCK-8; KeyGEN, Nanjing, China). The cells (1 × 10^3^) were seeded in 96-well plate and suffered with different drugs for 48 h, including ADR, paclitaxel, and vincristine (VCR, Sigma). In total 10 μl CCK-8 solution was added into per well at 37 °C and incubation for another 2 h. Absorbance at 450 nm (A450) was read on a microplate reader (168–1000 Model 680, Bio-Rad). The drug resistance was analyzed by comparing the IC_50_ values (the drug concentration that inhibits cell growth by 50%).

### Methylcellulose colony formation assay

Colony formation assay was carried out to measure the capacity of cell proliferation. Briefly, 1 × 10^3^ cells were seeded in six-well plates. The medium of per well was mixed with 1 mL of methylcellulose (MethoCult GF M3534), and 2 ml RPMI 1640 medium containing 10% FBS. After 7–10 days, the colony numbers were counted under a microscope.

### Oligonucleotide construction and dual luciferase assay

PCR production of ALG3 and LncRNA FTX were cloned into the expression vector pcDNA3.1 (Invitrogen). MiR-342 mimic, negative control oligonucleotides (miR-NC), miR-342 inhibitor, negative control oligonucleotide (NC inhibitor), small interfering RNA of FTX (siFTX), scramble siRNA of FTX (siSCR) were purchased from RiboBio (Guangzhou, China). The cells were seeded into 6-well plates and transfection was performed using Lipofectamine 3000 (Invitrogen). The transfection efficiency was assessed by qRT-PCR.

Cells were cultured overnight until 70–80% confluence. Next, cells were co-transfected with pcDNA3.1 FTX-wt, pcDNA3.1 FTX-mut, pcDNA3.1 ALG3-wt or pcDNA3.1 ALG3-mut was transfected into HEK-293T cells together with miR-342 mimic or the control, respectively. Lipofectamine 3000 (Invitrogen) was used for transfection. The transfected cells were collected for luciferase detection by the dual-luciferase reporter gene assay system (Promega, Madison, WI, USA). Data were shown as the mean value±SD and each experiment was performed thrice.

### RNA immunoprecipitation (RIP) assay

The Magna RIP^TM^ RNA Binding Protein Immunoprecipitation Kit (Millipore, Bedford, MA, USA) was utilized to perform RIP assay. Cells were collected and lysed under RIPA buffer containing a protease inhibitor cocktail and RNase inhibitor. RIP buffer containing magnetic bead conjugated with human anti-Ago2 antibody (Millipore) or mouse immunoglobulin G (IgG) was added into the cell extracts. The protein was digested with proteinase K and subsequently the immunoprecipitated RNA was obtained. The qRT-PCR assay was used to measure the purified RNA, which better illustrated the potential the binding targets.

The article "Aberrant mannosylation profile and FTX/miR-342/ALG3-axis contribute to development of drug resistance in acute myeloid leukemia" was retracted in 2020. Reasons: duplicated data; concerns about the data.

### Antitumor activity in xenograft model

The male nude mice (5-week old) were purchased from the Model Animal Research Institute of Nanjing University. In total 1 × 10^7^ cells were injected subcutaneously into the right flank of nude mouse. The mice were randomly divided into control and treatment groups. The treatment groups suffered 7 mg/kg ADR i.p. three times a week for 3 weeks. The mice were humanely killed and their tumors were photographed. The tumor volume was calculated. The Committee on the Ethics of Animal Experiments of Dalian Medical University supported the xenografts model in vivo.

### Immunohistochemistry (IHC)

Xenograft tumors were isolated and executed on paraffin-embedded sections. The slides were deparaffinized, rehydrated and immersed in 3% hydrogen peroxide for 10 min to block endogenous peroxidase. The primary anti ALG3 or Ki67 antibody (1:200, Abcam) was added to the sections at 4 °C for 12 h. The secondary streptavidin-HRP-conjugated antibody (1:1000, Santa Cruz Biotech) was subsequently stained for 1 h. Then the hematoxylin was used to counterstain the slides.

### Statistical analysis

Data were analyzed by SPSS 13.0 and presented as the mean±standard deviation (SD). Student’s *t*-test was utilized to identify the significance of difference of two groups, and one-way analysis of variance (ANOVA) was used for multiple groups. *P < 0.05 was considered to be statistically significant.

## Results

### *N*-Glycan profles of AML cell lines

Total *N*-glycans from U/A and U937 cells were released by PNGase F and were analyzed by MALDI-TOF MS. A total composition of 23 *N*-linked glycan was found from the U/A and U937 cells and summarized in Table 1. The *N*-glycans of each fraction in MS spectrum was detected in the *m/z* range 1000–4000 (Fig. 1a). Relative expression of *N*-glycan composition produced from three replicates is shown in Fig. 1b. Using an average-fold change of ≥1.5, six peaks discriminated the U/A and U937 cells. Peaks 1, 3, 4, 12, 14, and 18 were up-regulated in U/A. The peaks at 2, 5, 6, 11, and 23 were detected in the drug-resistant U/A cells. High-mannose-type *N*-glycans (peak 1, 4, 7, 12, and 16) were observed in U/A and U937 cells (Table 1). Furthermore, U/A cells showed higher incidence of additional significant peaks at 1, 4 and 12 (high-mannose *N*-glycans). Thus, MALDI-TOF MS analysis revealed that elevated high-mannose *N*-glycans were presented in MDR of AML.

The article "Aberrant mannosylation profile and FTX/miR-342/ALG3-axis contribute to development of drug resistance in acute myeloid leukemia" was retracted in 2020. Reasons: duplicated data; concerns about the data.

**Table 1:** High-mannose-type N-glycans were shown in U/A and U937 cells

Glycan number	Observed *m/z*		Chemical composition
	U/A	U937	
1	1579.793	1579.758	Man_2_+Man_3_GlcNAc_2_
2	1620.822		HexHexNAc+Man_3_GlcNAc_2_
3	1661.846	1661.837	HexNAc_2_+Man_3_GlcNAc_2_
4	1783.892	1783.843	Man_3_+Man_3_GlcNAc_2_
5	1824.924		Hex_2_HexNAc+Man_3_GlcNAc_2_
6	1865.951		HexHexNAc_2_+Man_3_GlcNAc_2_
7	1987.998	1987.936	Man_4_+Man_3_GlcNAc2
8	2009.995	2009.930	HexNAc_2_Fuc_2_+Man_3_GlcNAc_2_
9	2029.019	2029.025	Hex_3_HexNAc+Man_3_GlcNAc_2_
10	2040.026	2040.041	HexHexNAc_2_Fuc+Man_3_GlcNAc_2_
11	2070.052		Hex_2_HexNAc_2_+Man_3_GlcNAc_2_
12	2192.098	2192.048	Man_5_+Man_3_GlcNAc2
13	2244.139	2244.122	Hex_2_HexNAc_2_Fuc+Man_3_GlcNAc_2_
14	2274.159	2274.141	Hex_3_HexNAc_2_+Man_3_GlcNAc_2_
15	2315.165	2315.120	Hex_2_HexNAc_3_+Man_3_GlcNAc_2_
16	2396.197	2396.155	Man_6_+Man_3_GlcNAc_2_
17	2431.208	2431.150	Hex_2_HexNAc_2_NeuAc+Man_3_GlcNAc_2_
18	2519.273	2519.212	Hex_3_HexNAc_3_+Man_3_GlcNAc_2_
19	2764.376	2764.393	Hex_3_HexNAc_4_+Man_3_GlcNAc_2_
20	2792.367	2792.396	Hex_2_HexNAc_2_NeuAc_2_+Man_3_GlcNAc_2_
21	2880.453	2880.498	Hex_3_HexNAc_3_NeuAc+Man_3_GlcNAc_2_
22	2968.494	2968.457	Hex_4_HexNAc_4_+Man_3_GlcNAc_2_
23	3417.787		Hex_5_HexNAc_5_+Man_3_GlcNAc_2_

**Fig. 1:** *N*-glycan composition in AML cell lines. **a** MALDI-TOF MS spectra of permethylated *N*-glycans released from U/A and U937 cells, respectively. **b** Histograms of relative intensities of the differential *N*-glycan signals from the both cell lines were observed. **c** The lectin microarray further determined the differential expression of lectin between U/A and U937 cells. **d** FCM was used to detect the MAN-M, ConA and AAL lectin expression in AML cell lines

To identify the cell surface glycan profiles associated with U/A and U937 cells, a lectin microarray containing 56 lectins was conducted. Three (namely, MAN-M, ConA, and Jacalin) were found to show noticeably different extents of binding to different membrane proteins (Fig. 1c). MAN-M and ConA were specific for mannose, indicating that high mannose oligosaccharides on U/A cell surface might be critical for AML MDR development.

To further verify the lectin microarray results, all three positive and one negative bindings on the microarray were evaluated by FCM. As shown in Fig. 1d, the similar binding tendencies were observed with the results of lectin microarray, with the highest binding observed for MAN-M in U/A. As shown in Fig. 1e, the binding of T/A cells to MAN-M and ConA lectins was higher than that of THP-1 cells. Interestingly, the binding of M5/MDR patients to MAN-M and ConA lectins was also higher than that of M5 patients (Fig. S1). The observation indicated that differential expression of high-mannose *N*-glycans might associate to AML drug resistance.

The article "Aberrant mannosylation profile and FTX/miR-342/ALG3-axis contribute to development of drug resistance in acute myeloid leukemia" was retracted in 2020. Reasons: duplicated data; concerns about the data.

### Expressional profile of ALG family in AML patients and cell lines

The extent of high-mannose-type *N*-glycans depended on mannosyltransferases. In this study, the levels of ALG gene family in two adriamycin-resistant (ADR) cell lines compared to parent cell lines were analyzed by qRT-PCR. As shown in Fig. 2a, remarkable increase of ALG3, ALG4 and ALG11 mRNA was observed in U/A and T/A cell lines compared with those of drug-susceptible parental cells lines U937 and THP-1 (*p < 0.05). In addition, two parent cell lines showed higher level of ALG9 (*p < 0.05). No statistically significant differences were found in other ALG genes, while ALG2 gene was almost absent in two pairs of AML cell lines. The group of M5/MDR showed significantly elevated ALG3 expression compared to M5 group (Fig. 2b, *p < 0.05). The expression of ALG3 was further measured in human leukemia cell lines and PBMC from M5 patients. The level of ALG3 protein was up-regulated in ADR-resistant cell lines and M5/MDR group (Fig. 2c). The Kaplan-Meier method was used to analyze the association of ALG3 level with overall survival (OS) in AML patients. The results showed that OS of patients with high ALG3 expression significantly decreased (*p < 0.05; Fig. 2d). The result indicated that ALG3 displayed a potential clinical utility to monitor the progression of AML drug resistance.

**Fig. 2:** Differential expression of ALG gene family in AML cell lines and AML patients. **a** The differential expression of ALG gene family was detected in AML cell lines by qRT-PCR. **b** The ALG family levels were measured in AML patients by qRT-PCR. **c** The ALG3 level was determined by western blot. **d** Kaplan–Meier overall survival curves (OS) was observed based on ALG3 level. Data were the means±SD of triplicate determinants (*p < 0.05)

### ALG3 modulates the chemosensitivity of AML cells in vitro and in vivo

To elucidate the impact on the chemosensitivity of ALG3 involved in AML cell lines, ALG3 expression was down-regulated in U/A and T/A cell lines. As shown in Fig. 3a, the ALG3 was significantly decreased in ALG3 shRNA transfectant compared to control (*p < 0.05). Furthermore, the mannose levels detected by FITC-MAN-M and FITC-ConA lectins on the cell surface were reduced in U/A-ALG3 shRNA and T/A-ALG3 shRNA cell lines (Fig. 3b).

**Fig. 3:** Knockdown of ALG3 attenuated MDR of AML cell lines. **a** ALG3 expression was detected by qRT-PCR and western blot in AML cell lines transfected with ALG3 shRNA. **b** FCM was used to show the mannose levels by FITC-conjugated MAN-M and FITC-ConA on the cell surface of transfected AML cell lines. **c** The chemoresistance to ADR, VCR and Paclitaxel was detected in AML cell lines by CCK8 assays. **d** The IC_50_ values was calculated and presented. **e** The proliferative formation in response to different drugs of transfected AML cell lines were examined by colony-forming unit assay. **f** FCM showed the apoptosis of transfected AML cell lines in response to ADR, VCR and paclitaxel. **g** The key apoptosis related molecules were determined by western blot. **h** The tumor tissues of nude mice were presented and the volume was calculated on the 7, 14, 21, and 28 days. **i** Different tumor tissues were sectioned and stained with ALG3 and Ki67 by IHC staining. Data were the means±SD of triplicate determinants (*p < 0.05)

The proliferative capability of AML cell lines was further performed using CCK8 assay. Interestingly, when ALG3 knockdown cells were incubated in the presence of the chemotherapeutic agent ADR, VCR, and Paclitaxel, the knockdown cells demonstrated a reduced capability to proliferate compared with their control groups (Fig. 3c). The IC_50_ values were significantly decreased in U/A-ALG3 shRNA group and T/A-ALG3 shRNA group (Fig. 3d). The average size of colonies in ALG3 shRNA treated group was smaller than the untreated group. The number of colony after ALG3 shRNA transduction was also dramatically reduced (Fig. 3e). Moreover, shRNA targeting ALG3, significantly enhanced the ability of chemotherapy-induced apoptosis in AML cell lines (Fig. 3f). Apoptosis was also assessed by the appearance of caspase-3 cleavage after western blot. As shown in Fig. 3g, with drug treatment, ADR cell lines transfected with ALG3 shRNA expressed low caspase3 and PARP levels, and increased levels of cleaved caspase3 and cleaved PARP. To further assess the chemosensitivity to ADR in vivo, mouse xenograft studies were performed. In the ALG3 shRNA model, down-expression of ALG3 significantly inhibited tumor growth. In a further study in the ADR treatment ALG3 shRNA model, the primary tumor volume was decreased with ADR treatment, while the decrease was in a faster rate (Fig. 3h). As shown in Fig. 3i, the expression of ALG3 and Ki67 in xenograft tumor was also verified by IHC staining. Furthermore, the proliferation of U/A and T/A cells was also measured without drug treatment. The proliferative ability was assessed by CCK8 assay (Fig. S2A), colony-forming unit analysis (Fig. S2B) and xenograft studies (Fig. S2C). IHC staining was conducted to evaluate the ALG3 and Ki67 levels (Fig. S2D). In addition, ALG5 gene was chosen to validate that modulation of ALG5 showed no effect on the biological function of U/A cells (Figs. S3A-3D). This part identified ALG3 indeed affected drug resistance of AML cells.

The article "Aberrant mannosylation profile and FTX/miR-342/ALG3-axis contribute to development of drug resistance in acute myeloid leukemia" was retracted in 2020. Reasons: duplicated data; concerns about the data.

Transfection of U937 and THP-1 cell lines with ALG3 resulted in an increase of ALG3 level compared to mock (Fig. 4a). Using FITC-MAN-M and -ConA lectin hybridization, differential expression of mannose was observed in the four groups. As shown in Fig. 4b, the binding of U937/ALG3 and THP-1/ALG3 to MAN-M and ConA lectins was higher than the mock. Furthermore, overexpression of ALG3 promoted U937/ALG3 and THP-1/ALG3 cells proliferation and chemoresistance to ADR, VCR and Paclitaxel (Fig. 4c). The IC_50_ values showed similar tendency (Fig. 4d). Colony formation assay further proved U937/ALG3 and THP-1/ALG3 cell lines had a variable degree in response to chemotherapy (Fig. 4e). Moreover, the ADR, VCR, and Paclitaxel significantly increased apoptosis rate (Fig. 4f). As shown in Fig. 4g, treatment of parent cell lines with ADR, VCR or Paclitaxel, the levels of ALG3-induced caspase3 and PARP were up-regulated, and down-regulation of cleaved caspase3 and cleaved PARP levels. Next, the antitumor activity of ADR against ALG3-driven leukemia tumor growth in nude mice was also assessed. Mean of tumor volume was shown in U937/ALG3 tumor compared to the control, and in U937/ALG3+ADR tumor compared with the mock+ADR group. Furthermore, ADR treatment significantly reduced U937/ALG3 tumor growth (Fig. 4h). IHC staining was performed on tumors to indicate the expression of ALG3 and Ki67 in tumors (Fig. 4i). Without drug treatment, upregulation of ALG3 in U937 and THP-1 cells facilitated cell proliferation (Fig. S2E, S2F) and tumor growth in vivo (Fig. S2G). ALG3 level was extremely higher in the group bearing U937/THP-1-ALG3 cells than the control group. Enhanced Ki67 expression showed strongly tumor growth (Fig. S2H). Overexpressed ALG5 presented no effect on drug sensitivities of U937 cells (Figs. S3E-3H). These results clearly demonstrated that ALG3 was responsible for the overcoming cell MDR via regulating high-mannose-type *N*-glycans in AML cells.

**Fig. 4:** Upregulation of ALG3 promoted MDR of AML cells. **a** qRT-PCR and western blot were carried out to detect ALG3 expression of different treated AML cell lines. **b** The expression of FITC-MAN-M and FITC-ConA was determined by FCM. **c** The alteration of chemosensitivity to ADR, VCR and Paclitaxel was detected in AML cell lines by CCK8 assays. **d** The IC_50_ values were subsequently calculated. **e** Proliferation of treated AML cells was observed by colony formation assay with the mediation of methylcellulose. **f** The apoptosis rate was clarified with ADR, VCR and paclitaxel treatment by FCM. **g** Caspase3, cleaved caspase3, PARP and cleaved PARP levels were analyzed by western blot. **h** The tumor tissues of nude mice was recorded and shown. **i** ALG3 and Ki67 expression was observed by IHC staining. Data were the means±SD of triplicate determinants (*p < 0.05)

The article "Aberrant mannosylation profile and FTX/miR-342/ALG3-axis contribute to development of drug resistance in acute myeloid leukemia" was retracted in 2020. Reasons: duplicated data; concerns about the data.

### FTX is a direct target of miR-342 and positively regulates the expression of ALG3 in AML cells

Recently, ceRNA have generated substantial interest and have been reported in many cancers. Bioinformatic analysis predicts that miR-342 is closely associated with lnc-FTX. The expression level of miR-342 was examined using qRT-PCR in two pairs of AML cell lines (Fig. 5a). Furthermore, the miR-342 was expressed at lower level in the M5/MDR group compared with M5 group (*p < 0.05, Fig. 5b), indicating that miR-342 was frequently down-regulated in AML MDR. A significant negative correlation was observed between miR-342 and ALG3 mRNA (*r* = −0.5828, *p* < 0.0001, Fig. 5c) in PBMC of AML patients. We examined the seed sequence of miR-342 in ALG3 and found a predicted binding site for miR-342 (Fig. 5d). Dual-luciferase reporter gene assay confirmed that ALG3 was a direct target of miR-342 (Fig. 5d). U/A and T/A cells were transiently transfected with miR-342 mimic or inhibitor to study the effect of miR-342 on ALG3 expression. MiR-342 mimic significantly decreased expression of ALG3 (Fig. 5e). MiR-342 inhibitor also increased ALG3 expression (Fig. 5f). These results indicated a strong inverse correlation between expression of ALG3 and miR-342.

**Fig. 5:** FTX directly bound miR-342 and regulated ALG3 expression. **a** The miR-342 expression was determined in AML cell lines by qRT-PCR. **b** The level of miR-342 was then detected in M5/MDR patients and M5 patients groups. **c** The correlation between ALG3 and miR-342 was determined by Spearman’s correlation analysis. **d** Sequence aligment of miR-342 with predicted binding sites in the wild-type and mutant-type regions of ALG3 (left panel) was shown. **e** The ALG3 expression was shown with miR-342 mimic treated AML cell lines. **f** The ALG3 expression was shown with miR-20b inhibitor treated AML cell lines. **g** FTX levels of AML cell lines were determined by qRT-PCR. **h** qRT-PCR was used to analyze the FTX expression in AML patients. **i** The Spearman’s correlation was used to analyze the relationship between FTX and miR-342 expression. **j** Sequence aligment of miR-342 with putative binding sites in the wild-type and mutant-type regions of FTX (left panel) was shown. The wild-type and mutant miRNA target FTX sequences were fused with luciferase reporter, transfected with miRNA mimic and NC mimic (right panel). **k**, **l** The FTX expression was detected in AML cell lines with miR-342 mimic and inhibitor treatment by qRT-PCR. **m**, **n** The ALG3 level was determined in AML cell lines with different treatment of FTX. **o** The co-precipitated RNA was detected by qRT-PCR in RNA immunoprecipitation experiment. FTX and miR-342 were presented as fold enrichment in Ago2 relative to IgG immunoprecipitate. Data were the means±SD of triplicate determinants (*p < 0.05)

To further determine whether FTX actually bound with miR-342, FTX level was measured by qRT-PCR in AML cells. FTX expression was higher in ADR-resistant AML cell lines than primary cells (Fig. 5g). FTX was also more highly expressed in M5/MDR group compared with M5 group (*p < 0.05, Fig. 5h). Pearson correlation coefficient analysis showed a negative correlation between FTX and miR-342 in PBMC of AML patients (Fig. 5i). Furthermore, cells transfected with wt-FTX and the miR-342 mimic revealed lower luciferase intensity compared to other groups (Fig. 5j), confirming that FTX was a direct target of miR-342. MiR-342 mimic decreased the FTX level in U/A and T/A cells (Fig. 5k). In contrast, anti-miR-342 dramatically up-regulated FTX expression in U937 and THP-1 cells (Fig. 5l), which indicated miR-342 could be a negative regulator of FTX. In U937 and THP-1 cells, siFTX reduced ALG3 expression, whereas overexpression of FTX induced ALG3 expression, indicating that positively regulated ALG3 expression (Fig. 5m, n).

The article "Aberrant mannosylation profile and FTX/miR-342/ALG3-axis contribute to development of drug resistance in acute myeloid leukemia" was retracted in 2020. Reasons: duplicated data; concerns about the data.

To further verify whether FTX associated with miRNP, RNA binding protein immunoprecipitation (RIP) assay was performed on AML cell line extracts using anti-Ago2 antibody. FTX and miR-342 were significantly enriched in Ago2- containing immunoprecipitate compared with control immunoglobulin G (IgG) immunoprecipitate (Fig. 5o), confirming the association of FTX and miR-342. Thus, FTX functioned as a competing endogenous RNA to regulate ALG3 level by sponging miR-342 in AML cell lines.

### FTX and miR-342 modulate ADR resistance of AML cells through regulating ALG3 expression

To investigate the relationships among FTX, miR-342 and ALG3 and their effects on the MDR development of AML, U/A and T/A cells were transfected with siFTX or siSCR, anti-miR-342 or anti-miR-NC. Compared with control, the ALG3 mRNA level was significantly up-regulated by anti-miR-342 and was down-regulated by siFTX (Fig. 6a, *p < 0.05). Co-transfection of anti-miR-342 and siFTX showed that anti-miR-342 partially restored the suppression of ALG3 level by siFTX (Fig. 6a, lane 4 compared with lane 3, respectively). Similar results were also detected by western blot in AML cell lines (Fig. 6b). As shown in Fig. 6c, anti-miR-342 promoted the mannose levels (detected by FITC-MAN-M and FITC-ConA lectins) on the cell surface compared to negative control. The mannose levels were down-regulated after FTX knockdown. More importantly, anti-miR-342 partially reversed the decreased mannose level induced by siFTX. Furthermore, the potential function of FTX-miR-342 pathway to ADR resistance was evaluated. The U/A and T/A cells became resistant to ADR after anti-miR-342, while cells transfected with siFTX remained sensitive to ADR. Anti-miR-342 attenuated the cell sensibility to ADR induced by siFTX (Fig. 6d). The IC_50_ values showed similar tendency (Fig. 6e). Treatment with ADR, colony-forming assay data revealed that anti-miR-342 promoted U/A and T/A cell growth, whereas siFTX inhibited cell growth after ADR treatment. Co-transfection of anti-miR-342 and siFTX expression plasmid showed that anti-miR-342 promoted the proliferation suppressed by siFTX (Fig. 6f). Treatment with ADR, anti-miR-342 reduced cell apoptosis, whereas siFTX promoted apoptosis (Fig. 6g). Co-transfection of anti-miR-342 and siFTX showed that anti-miR-342 restored apoptosis promoted by siFTX.

The article "Aberrant mannosylation profile and FTX/miR-342/ALG3-axis contribute to development of drug resistance in acute myeloid leukemia" was retracted in 2020. Reasons: duplicated data; concerns about the data.

**Fig. 6:** The reversal effort of co-expreesion siFTX and anti-miR-342 on AML chemoresistance. **a** ALG3 expression was detected by qRT-PCR with co-transfection siFTX and anti-miR-342 in AML cell lines. **b** Western blot was used to detect ALG3 level in AML cell lines. **c** FCM showed altered mannose level of different treated AML cell lines through FITC-MAN-M and FITC-ConA. **d** The viability of AML cells was detected by CCK8 with ADR treatment. **e** The altered IC_50_ values were calculated. **f** With ADR treatment, the colony formation ability was determined. **g** FCM showed the apoptosis rate of transfected AML cells in response to ADR. Data were the means±SD of triplicate determinants (*p < 0.05)

ALG3 were down-regulated by miR-342 mimic in U937 and THP-1 cells, whereas FTX overexpression enhanced ALG3 level. Co-transfection of FTX and miR-342 showed that miR-342 partially abrogated the increase in ALG3 level by FTX, suggesting that FTX regulated the miR-342 target gene ALG3 (Fig. 7a, b). As shown in Fig. 7c, altered mannose-type *N*-glycans in AML cell lines were revealed by fluorescence intensity on FITC-MAN-M and FITC-ConA lectins. MiR-342 mimic inhibited U937 and THP-1 cell growth after ADR treatment (Fig. 7d). Interestingly, up-regulated FTX promoted the growth of U937 and THP-1 cells, and this growth could be reversed by miR-342 mimic. Furthermore, the IC_50_ of ADR on AML cell lines was detected (Fig. 7e). A corresponding effect on colony-formation abilities was also observed in a parallel clonogenic assay, further supporting the role of FTX and miR-342 in mediating ADR-resistant cell growth (Fig. 7f). Finally, cell apoptosis induced by FTX or miR-342 in U937 and THP-1 cells was detected by FCM (Fig. 7g). In short, all the outcomes above explained the function and regulatory mechanism of FTX/miR-342/ALG3 axis in the development of AML drug resistance.

The article "Aberrant mannosylation profile and FTX/miR-342/ALG3-axis contribute to development of drug resistance in acute myeloid leukemia" was retracted in 2020. Reasons: duplicated data; concerns about the data.

**Fig. 7:** The reversal effect of co-expreesion FTX and miR-342 on AML chemoresistance. **a** qRT-PCR was carried out to detect ALG3 expression in the transfected AML cell lines. **b** ALG3 level was determined by western blot. **c** FITC-MAN-M and FITC-ConA were detected by FCM to show the mannose level of transfected AML cell surface. **d** With ADR treatment, the cell viability was determined by CCK8 assay. **e** The IC_50_ values of transfected AML cell lines were calculated and presented. **f** The proliferative ability was observed in response to ADR treatment. **g** The apoptosis induced by ADR was determined by FCM. Data were the means±SD of triplicate determinants (*p < 0.05)

## Discussion

*N*-linked glycans have been shown to change in the malignant phenotype of cancer cells and drug-resistance potential. Drawing the altered patterns of *N*-glycans enriches our understanding on the molecular mechanism of glycosylation in AML drug-resistance. Analysis of *N*-glycans by MALDI-TOF MS represents a new paradigm in cancer biomarker studies. In this work, the *N*-linked glycans were monitored during the drug-resistance of AML cells. Our analysis of *N*-glycans released from total membrane glycoproteins demonstrated unexpected diversity of *N*-glycans between U/A and U937 cell lines by MS. The detected changes in glycan expression were also correlated with drug-resistance in AML. The result was in accordance with our previous reports on the differential *N*-glycan profiles between leukemia K562/ADR cells and K562 cells, HL60/ADR and HL60 cells^19,20^. Moreover, major peaks (the peaks at 1, 4, and 12) corresponded to high-mannose type *N*-glycans originating from U/A cells also showed an increase. The elevation of high-mannose glycans was consistent with other reports that correlated their behavior with cancer^21^. Another report showed that cisplatin-resistant KCP-4 cells from KB-3-1 human carcinoma exhibited an increase in the high-mannose glycans^22^. In addition, lectin microarray of U/A and U937 cells revealed differential expression of mannose (recognized by MAN-M and ConA, respectively), which were further evaluated by FCM. This suggested that high-mannose *N*-glycan alteration might be AML drug resistance-specific. This drug resistance-specific made high-mannose glycans more promising as a potential biomarker for early diagnosis of drug resistance in AML.

The article "Aberrant mannosylation profile and FTX/miR-342/ALG3-axis contribute to development of drug resistance in acute myeloid leukemia" was retracted in 2020. Reasons: duplicated data; concerns about the data.

Differential expression of glycosyltransferases within the tumor cell is one of the primary causes of aberrant glycosylation in cancer^6^. ALG family represent an important group of glycosyltransferases. The expression profiles of ALG gene family were differed in AML cell lines and AML samples. ALG3, which encodes an alpha-1, 3-mannosyltransferase involved in the build-up of dolichol linked high-mannose type glycans in the ER^23^. Elevated levels of ALG3 have been observed in MDR cell lines and PBMC of M5/MDR patients. ALG3 mRNA expressed at highest level that conferred to the high level of high-mannose glycans (Man_6_GlcNAc_2_) on U/A cell surface. This was consistent with previous reports that ALG3 expression was higher in esophageal squamous cell carcinoma, especially in patients with lymph node metastasis^24^, and high level of ALG3 was significantly correlated with cervical cancer^25^. Interestingly, increased ALG3 level was also associated with OS in AML patients. ALG9 gene, encoding alpha-1, 2-mannosyltransferase, participated in the formation of the lipid-linked oligosaccharide precursor of *N*-glycosylation^26^. The pathogenic variants in ALG9 could present as a lethal skeletal dysplasia with visceral malformations^27^. In this study, significant reduced ALG9 was observed in MDR cell lines and PBMC of M5/MDR patients, which was accompanied with an accumulated both ALG9 substrates Man_6_GlcNAc_2_ and Man_8_GlcNAc_2_. In agreement with this observation, cells lacking ALG9 accumulated Man_6_GlcNAc_2_ and Man_8_GlcNAc_2_^27^. In addition, altered ALG3 (responsible for mannosylation) has been associated with drug resistance of AML cells, supporting the functional involvement of mannosylation in AML chemotherapy processes. Thus, the ability to distinguish the differences in the mannosylation and mannosyltransferases between AML parent and MDR cell lines underscored glycobiology as a promising field for identification of potential AML biomarkers.

In recent years, the ceRNA model was proposed, indicating that abundant cytoplasmic lncRNAs could interact with miRNAs seed sequences through miRNA-binding sites to reduce their regulatory effect on target mRNA, the so-called miRNA sponge^28^. MiRNAs also played an important role in the ceRNA network through combining with target mRNA, inhibiting the action of mRNA expression^29^. Plasma level of miR-342 was significantly down-regulated in the AML patients in comparison with control group^30^. MiR-342 regulated tamoxifen response in breast tumor cell lines^31^. LncRNA FTX contributed to tumor progression through mechanism including ceRNA has generated substantial interest and has been reported in many cancers^32,33^. FTX was highly expressed in gliomas and was critical for glioma cell proliferation and invasion by regulating miR-342-3p and AEG-1^34^. In this study, we found that FTX expression was inversely correlated to miR-342 level in AML cell lines and AML patients. MiR-342 bound to FTX in a sequence-specific manner and regulated FTX expression. On the other hand, miR-342 expression was negatively correlated with ALG3. Moreover, ALG3 was a direct target of miR-342 and could be modulated by miR-342. In addition, both FTX and miR-342 were associated with the immunoprecipitated Ago2 complex, and the Ago2 complex cleaved FTX in the presence of miR-342 in AML cell lines. Interestingly, we also revealed that altered FTX and miR-342 was significantly associated with ALG3 expression, and lectins (MAN-M and ConA) exhibited a different degree of consistency in AML cell lines. Knockdown of FTX inhibited the drug resistance of AML cell lines to ADR, while miR-342 inhibitor restored the impact on chemosensitivity exerted by FTX inhibition. These results provided convincing evidence regarding the reciprocal repression loop of FTX/miR-342/ALG3 in a functional aspect.

The article "Aberrant mannosylation profile and FTX/miR-342/ALG3-axis contribute to development of drug resistance in acute myeloid leukemia" was retracted in 2020. Reasons: duplicated data; concerns about the data.

In conclusion, the present study provides evidence, for the first time, that mannosyltransferases and mannosylation may play important roles in the ADR resistance in AML cell lines. However, the mechanisms of ADR resistance in AML may be multifactorial. Dysregulated expression of FTX may function as the endogenous sponge to regulate ALG3 level by competitively binding miR-342 in AML cells. The present study provides useful information to find new biomarkers for early diagnosis and therapeutic application in AML resistance.

## Electronic supplementary material

Figure S1

Figure S2

Figure S3

Table S1

## References

[1] Dohner H, Weisdorf DJ, Bloomfield CD (2015). Acute myeloid leukemia. N. Engl. J. Med..

[2] Burnett A, Wetzler M, Lowenberg B (2011). Therapeutic advances in acute myeloid leukemia. J. Clin. Oncol..

[3] Dube DH, Bertozzi CR (2005). Glycans in cancer and inflammation–potential for therapeutics and diagnostics. Nat. Rev. Drug. Discov..

[4] Pinho SS, Reis CA (2015). Glycosylation in cancer: mechanisms and clinical implications. Nat. Rev. Cancer.

[5] Hakomori S (1989). Aberrant glycosylation in tumors and tumor-associated carbohydrate antigens. Adv. Cancer Res..

[6] Meany DL, Chan DW (2011). Aberrant glycosylation associated with enzymes as cancer biomarkers. Clin. Proteom..

[7] Drake RR (2015). Glycosylation and cancer: moving glycomics to the forefront. Adv. Cancer Res..

The article "Aberrant mannosylation profile and FTX/miR-342/ALG3-axis contribute to development of drug resistance in acute myeloid leukemia" was retracted in 2020. Reasons: duplicated data; concerns about the data.

[8] Stowell SR, Ju T, Cummings RD (2015). Protein glycosylation in cancer. Annu. Rev. Pathol..

[9] de Leoz ML (2011). High-mannose glycans are elevated during breast cancer progression. Mol. Cell. Proteom..

[10] Chik JH (2014). Comprehensive glycomics comparison between colon cancer cell cultures and tumours: implications for biomarker studies. J. Proteom..

[11] Machova Polakova K (2011). Expression patterns of microRNAs associated with CML phases and their disease related targets. Mol. Cancer.

[12] Saki N, Abroun S, Hajizamani S, Rahim F, Shahjahani M (2014). Association of chromosomal translocation and MiRNA expression with the pathogenesis of multiple myeloma. Cell J..

[13] Zhu C (2013). Prognostic value of miR-29a expression in pediatric acute myeloid leukemia. Clin. Biochem..

[14] Lu F (2014). miR-181b increases drug sensitivity in acute myeloid leukemia via targeting HMGB1 and Mcl-1. Int. J. Oncol..

[15] Kung JT, Colognori D, Lee JT (2013). Long noncoding RNAs: past, present, and future. Genetics.

[16] Huarte M (2015). The emerging role of lncRNAs in cancer. Nat. Med..

[17] Xing CY (2015). Long non-coding RNA HOTAIR modulates c-KIT expression through sponging miR-193a in acute myeloid leukemia. FEBS Lett..

[18] Diaz-Beya M (2015). The lincRNA HOTAIRM1, located in the HOXA genomic region, is expressed in acute myeloid leukemia, impacts prognosis in patients in the intermediate-risk cytogenetic category, and is associated with a distinctive microRNA signature. Oncotarget.

[19] Zhang Z (2012). Glycomic alterations are associated with multidrug resistance in human leukemia. Int. J. Biochem. Cell. Biol..

[20] Ma H (2015). Modification of sialylation is associated with multidrug resistance in human acute myeloid leukemia. Oncogene.

[21] Lattova E, Tomanek B, Bartusik D, Perreault H (2010). N-glycomic changes in human breast carcinoma MCF-7 and T-lymphoblastoid cells after treatment with herceptin and herceptin/Lipoplex. J. Proteome Res..

[22] Nakagawa H (2008). Alterations in the glycoform of cisplatin-resistant human carcinoma cells are caused by defects in the endoplasmic reticulum-associated degradation system. Cancer Lett..

[23] Henquet M (2008). Identification of the gene encoding thealpha1,3-mannosyltransferase (ALG3) in Arabidopsis and characterization of downstream n-glycan processing. Plant Cell.

[24] Shi ZZ (2014). Identification of putative target genes for amplification within 11q13.2 and 3q27.1 in esophageal squamous cell carcinoma. Clin. Transl. Oncol..

[25] Choi YW (2007). Gene expression profiles in squamous cell cervical carcinoma using array-based comparative genomic hybridization analysis. Int. J. Gynecol. Cancer..

The article "Aberrant mannosylation profile and FTX/miR-342/ALG3-axis contribute to development of drug resistance in acute myeloid leukemia" was retracted in 2020. Reasons: duplicated data; concerns about the data.

[26] Tham E (2016). A novel phenotype in N-glycosylation disorders: Gillessen-Kaesbach–Nishimura skeletal dysplasia due to pathogenic variants in ALG9. Eur. J. Human. Genet..

[27] Frank CG, Aebi M (2005). ALG9 mannosyltransferase is involved in two different steps of lipid-linked oligosaccharide biosynthesis. Glycobiology.

[28] Quinn JJ, Chang HY (2016). Unique features of long non-coding RNA biogenesis and function. Nat. Rev. Genet..

[29] Bartel DP (2009). MicroRNAs: target recognition and regulatory functions. Cell.

[30] Elhamamsy AR (2017). Circulating miR-92a, miR-143 and miR-342 in plasma are novel potential biomarkers for acute myeloid leukemia. Int. J. Mol. Cell Med..

[31] Cittelly DM (2010). Downregulation of miR-342 is associated with tamoxifen resistant breast tumors. Mol. Cancer.

[32] Liu F (2016). Long noncoding RNA FTX inhibits hepatocellular carcinoma proliferation and metastasis by binding MCM2 and miR-374a. Oncogene.

[33] Liu Z (2016). Ftx non coding RNA-derived miR-545 promotes cell proliferation by targeting RIG-I in hepatocellular carcinoma. Oncotarget.

[34] Zhang W (2017). Long noncoding RNA FTX is upregulated in gliomas and promotes proliferation and invasion of glioma cells by negatively regulating miR-342-3p. Lab. Investig..

